The article "Effects of Chinese Herbal Formula on Immune Function and Nutritional Status of Breast Cancer Patients" was retracted in 2023. Reasons: unreliable results or conclusions; concerns about the data; concerns about the peer review; concerns about the citations.

# Effects of Chinese Herbal Formula on Immune Function and Nutritional Status of Breast Cancer Patients

**DOI:** 10.1155/2022/5900024

**Published:** 2022-07-14

**Authors:** Min Liu

**Affiliations:** Department of Clinical Nutrition, Affiliated Hospital of Shandong University of TCM, Jinan 250011, China

## Abstract

**Background:**

Chinese herbal formulas have certain effects on patients with breast cancer (BC). This article discussed the effect of Buqi Yangxue decoction on the immune function and nutritional status of BC patients and provided an evidence for traditional Chinese medicine (TCM) to improve the quality of life and curative effect of BC patients.

**Methods:**

66 cases of BC patients were divided into control group (*n* =33) and Chinese herbal formula group (*n* =33). The control group was received with TE chemotherapy, and the Chinese herbal formula group was received with Buqi Yangxue decoction combined with TE chemotherapy. Nutritional status, immune function, TCM symptom quantitative score, and adverse reactions were compared between the two groups.

**Results:**

There was no difference in all indexes between the two groups before intervention. After 4 weeks, the nutritional indexes ALB, PA, TRF, and TP in Chinese herbal formula group were higher than those in control group, except HGb. CD3+, CD4+, and CD4+/CD8+ in both groups were sharply higher than before treatment, while CD8+ was dramatically lower, and the changes in Chinese herbal formula group were more obvious than those in control group. In Chinese herbal formula group, the levels of IgG, IgA, and IgM were sharply increased compared with control group. The TCM syndrome scores in both groups were decreased significantly after treatment, especially in Chinese herbal formula group. In addition, nausea and vomiting, inappetence, liver function impairment, leukopenia, and thrombocytopenia occurred in both groups. There was no clear difference in the incidence of adverse reactions between Chinese herbal formula group and control group.

**Conclusion:**

Buqi Yangxue decoction can effectively improve the nutritional status and immune function of BC patients, which has important clinical significance for the later comprehensive treatment.

## 1. Introduction

Breast cancer (BC) is one of the most common malignant tumors that seriously endangers women's health and life. In recent years, with environmental pollution, the change of people's lifestyle, and the increase of competitive pressure, the incidence of BC is increasing year by year [1, 2]. The incidence of BC in western developed countries accounts for the first place of female malignant tumors [3]. The incidence of BC has increased significantly in China, and the onset age is gradually becoming younger [4]. BC has surpassed cervical cancer and become the most common malignant tumor in urban women. Sadly, BC is becoming younger and younger, which seriously endangers the physical, mental health, and life safety of young women.

The main treatment for BC is surgical resection and postoperative chemotherapy [5, 6]. The depression, damage of qi and blood, hematocele, and fluid accumulation of postoperative BC patients affect the wound healing and body repair [7]. BC patients' weak constitution, combined with the toxic damage of surgical chemoradiotherapy drugs, makes their vital qi more weak. The immune function of patients with BC is generally low [8]. Immune system plays a very important role in reducing postoperative complications and preventing and limiting the occurrence and development of tumors [9]. The postoperative immune function of patients with BC is low, which will increase the risk of infection and tumor recurrence. Therefore, it is very important to restore the patient's immune function as soon as possible. However, due to the damage to the human immune system after treatment, as well as the depression of patients, it will inevitably lead to insufficient nutritional intake of patients. Persistent nutritional deficiencies can further affect recovery and treatment [10].

In the comprehensive treatment of BC, Chinese herbal formulas play a positive role in increasing curative effect, enhancing physical fitness, improving life quality, and alleviating side effects [11, 12]. Surgery and chemotherapy are the methods of removing evil, which are easy to harm the patient's vital qi, resulting in more deficiency of the patient's vital qi. Malignant tumors belong to qi and blood deficiency syndrome, and massive blood loss caused by surgery will lead to aggravation of qi and blood deficiency [13]. Therefore, BC patients should be treated with Chinese herbal formula during the treatment to achieve the effect of nourishing and eliminating pathogenic factors. In recent years, the basic principle of TCM in treating BC is to replenish T qi and blood. Lee et al. found that Huanglian Wendan Tang improved the prognosis of BC patients [14]. Moreover, Yanghe decoction was found to improve the immune function of BC patients [15]. Buqi Yangxue decoction is a famous prescription for treating deficiency of qi and blood. In recent years, with the application of modern research technology, the pharmacological action of this decoction has been further studied. Studies have shown that Buqi Yangxue decoction can promote the treatment of renal anemia [16]. Furthermore, Buqi Yangxue decoction improved TCM clinical symptoms of patients with advanced colorectal cancer, reduced the side effects of chemotherapy, and provided patients with quality of life [17].

In this study, 66 patients with BC were treated with Buqi Yangxue decoction adjuvant therapy, in order to provide theoretical basis for the study of Chinese herbal formulas to improve the therapeutic effect of BC patients.

## 2. Materials and Methods

### 2.1. Clinical Data and Methods

A total of 66 patients with BC from December 2019 to January 2021 were selected as the study subjects. Patients were divided into the control group and Chinese herbal formula group by numerical randomization. There were no significant differences in age, weight, tumor site, TNM stage, and lymph node metastasis between the two groups (Table 1, *P* > 0.05). All patients were clearly diagnosed with BC by preoperative biopsy or intraoperative pathological section. This study was approved by the Hospital's Ethics Committee. All patients were aware of the study and had signed informed consent.

### 2.2. Inclusion Criteria

1. Diagnosed with breast cancer by cytology and histopathology
2. No other malignant tumors
3. The expected survival was greater than 6 months
4. Those who agree to participate in the study and sign the informed consent

### 2.3. Exclusion Criteria

1. Concurrent use of drugs affecting the results of this study
2. Failure to follow the prescribed medication
3. With heart, liver, kidney, and other serious diseases
4. Mental disorders, unable to cooperate with evaluators

### 2.4. Interventions

The control group was treated with TE chemotherapy, and received routine nutritional intervention measures. Patients were given targeted dietary guidance according to the actual situation, chose light, digestible, and nutritious food, and avoided spicy stimulation and raw, cold, and greasy food.

The Chinese herbal formula group was treated with Buqi Yangxue decoction on the basis of the control group. The decoction was as follows: 15 g of Astragali Radix, 12 g of Codonopsis Radix, 10 g of Polygonati Rhizoma, 15 g of Rehmanniae Radix Praeparata, 10 g of Poria, 12 g of Radix Paeoniae Alba, 15 g of Angelica sinensis, 15 g of Chinese date, 6 g of liquorice. These herbs were decocted to 300 ml in water and taken twice in the morning and evening once a day, and taken continuously for 4 weeks.

### 2.5. Nutritive Indexes

In both groups, fasting venous blood was taken in the morning. The levels of hemoglobin (HGb), serum albumin (ALB), prealbumin (PA), transferrin (TRF), and serum total protein (TP) were measured by an automatic biochemistry analyzer (Cobas c702, Roche, Switzerland).

### 2.6. Cellular Immune Function Detection

Fasting venous blood was collected to detect various immune function indexes. CD3+, CD4+, CD8+, and CD4+/CD8+ were measured by flow cytometry (BeckMan Coulter). Peripheral blood immunoglobulin (IgA, IgG, and IgM) concentration was detected by radioimmunoassay.

### 2.7. TCM Syndrome Score

TCM syndrome score of patients was evaluated according to the Guidelines for Clinical Research of TCM New Drugs. The main symptoms were fatigue, self-care ability, nausea and vomiting, dizziness, loss of appetite, and insomnia. Symptoms were rated from 0 to 6 on a scale of severity. The score was 0 for no symptoms, 2 for mild symptoms, 4 for moderate symptoms, and 6 for severe symptoms. The total score was 0-36, with a lower score indicating a milder disease.

### 2.8. Adverse Reactions

The adverse reactions of BC patients in two groups during treatment were observed and recorded, including nausea and vomiting, loss of appetite, thrombocytopenia, leukopenia, and liver function damage.

### 2.9. Statistical Analysis

SPSS 24.0 was used to analyze and process the data. *t* test was used for measurement data analysis, and *χ*^2^ test was used for counting data analysis. *P* < 0.05 indicated that the difference was statistically significant.

## 3. Results

### 3.1. Comparison of Nutritional Indexes between the Two Groups

There was no significant difference in nutritional indexes between the two groups before the intervention. After 4 weeks, the nutritional indexes ALB, TP, PA, and TRF in Chinese herbal formula group were superior to the control group, except HGb (Table 2). Our results indicated that Buqi Yangxue decoction can dramatically improve the nutritional status of BC patients.

### 3.2. Comparative Analysis of Immune Function between the Two Groups

After treatment, CD3+, CD4+, CD4+/CD8+ were significantly increased, and CD8+ was significantly decreased in Chinese herbal formula group and control group (Table 3). And the changes of T lymphocytes in Chinese herbal formula group were clearly higher than that of control group after treatment. There was no obvious difference in the levels of immune indexes (IgG, IgA, and IgM) in both groups before intervention (Table 4). After treatment, the levels of serum IgG, IgA, and IgM in Chinese herbal formula group were notably higher than those in control group. Therefore, the data indicated that Buqi Yangxue decoction might improve the immune function of BC patients.

### 3.3. Comparison of TCM Symptom Quantitative Score between the Two Groups

Before treatment, there was no difference in observation symptom quantitative score between the two groups. After 4 weeks of treatment, observation symptom quantitative evaluation scale score in Chinese herbal formula group was notably lower than that in control group (Table 5). Our results manifested that Buqi Yangxue decoction might be helpful to improve the clinical symptoms of BC patients.

### 3.4. Comparison of Adverse Reactions between the Two Groups

Adverse reactions were found to be occurred in both groups during treatment, including nausea and vomiting, inappetence, liver function impairment, leukopenia, and thrombocytopenia. Results of Table 6 showed that there was no clear difference in the incidence of adverse reactions between the Chinese herbal formula group and control group. Therefore, our results indicated that Buqi Yangxue decoction was safe for the treatment of BC.

## 4. Discussion

BC is a common malignant tumor in women, and its exact pathogenesis has not been clarified yet. TCM believes that deficiency of vital qi and deficiency of blood is the internal cause and root of BC [18]. “Vital qi” in TCM is the immune function of modern medicine. The basis of the occurrence of malignant tumors is the weakness of vital qi, which is manifested in the low immune function. In TCM, the method of “Fuzheng cultivation” is adopted, which is to improve the immune function of the body by tonifying the innate kidney essence and the acquired spleen and stomach [19]. In the process of disease progression, patients often have deficiency syndromes such as spleen and stomach weakness, deficiency of qi and blood, depletion of yang qi, kidney failure, and deficiency of essence. Therefore, the method of replenishing qi and nourishing blood should run through the treatment process of BC [20]. Researches have shown that Chinese medicine has played an important role in the treatment of BC. Chinese herbal formula can be used as a complementary therapy, combined with surgery, chemotherapy, or targeted therapy, to enhance the immune function of patients and reduce adverse reactions [21, 22].

In this study, on the basis of conventional treatment, Buqi Yangxue decoction was used. Astragali Radix [23] and Poria [24] can obviously enhance and regulate the immune function of the body. Codonopsis Radix can tonify and replenish the middle qi, and nourish the heart to tranquilize [25]. Angelica sinensis and Rehmanniae Radix Praeparata have the function of promoting blood circulation and replenishing blood [26]. Polygonati Rhizoma can invigorate qi and nourish Yin [27]. Radix Paeoniae Alba can nourish blood and liver [28]. All the above herbs can nourish and replenish blood, and play the role of replenishing both qi and blood. Combined with licorice and Chinese date can soothe the liver and regulate qi, harmonize the spleen and stomach, and nourish qi and yin [29, 30]. All herbs are used together to play the effect of regulating qi and relieving depression, nourishing blood, and supplementing qi.

Immunosuppressant factors will be secreted or produced during the occurrence and development of tumors, so the immune function of patients with advanced malignant tumors is mostly in a suppressed state, which is the “deficiency of vital qi” in TCM. When the body is lack of vital qi, it will lead to the decline of “zang fu” function over time, and the resistance to disease will also be reduced. The occurrence and development of diseases are closely related to the changes in the number, function, activity, and proportion of CD3+,CD4+ and CD8+ cells [31]. Measuring the changes of CD3+, CD4+, CD4+/ CD8+ can directly reflect the immune function [32, 33]. CD3+ and CD4+ cells were significantly increased in Chinese herbal formula group, while CD8+ cell subsets were decreased, indicating that the cellular immune function of patients was improved. IgG, IgA, and IgM are important indexes of humoral immune response [34]. The results of this study showed that Buqi Yangxue decoction notably increased the levels of IgG, IgA, and IgM, indicating that it can improve the immune function of BC patients.

In addition, the study found that ALB, PA, TRF, and TP in the Chinese herbal formula group were clearly higher than those in the control group, which indicated that Buqi Yangxue decoction could improve the nutritional status of BC patients. Malnutrition in BC patients affects not only the immune system but also the patient's ability to tolerate treatment. Therefore, BC patients should strengthen nutrition during treatment to improve the therapeutic effect. Furthermore, Buqi Yangxue decoction was discovered to improve the TCM symptom. Ultimately, there was no significant difference in the incidence of adverse reactions between the two groups, suggesting that Buqi Yangxue decoction can be safely used for adjuvant treatment of BC.

To be sure, there are still some shortcomings in our research. For example, the number of experimental patients should be increased to ensure the accuracy of the experiment. The research method was simple and research indicators were few. Furthermore, the observation period was short, and the decoction for Buqi Yangxue decoction should be taken for a long time to verify its effect on BC. In addition, we should study the mechanism of Buqi Yangxue decoction in treating BC patients from the perspective of molecular biology.

## 5. Conclusion

To sum up, Buqi Yangxue decoction can improve the immune function, nutritional status, and TCM symptoms of BC patients, and with fewer adverse reactions. Our results may provide a new idea for the clinical treatment of BC with combination of Chinese and Western medicine.

## Figures and Tables

**Table 1:** Comparison of general data between the two groups before treatment.

	Chinese herbal formula group	Control group	*P*
Average age (years)	56.62 ± 8.26	57.23 ± 8.21	>0.05
Weight (kg)	50.37 ± 6.12	49.54 ± 7.15	>0.05
Tumor site			>0.05
Left	12	10	
Right	11	13	
TNM stage			>0.05
I-II	9	8	
III-IV	14	15	
Lymph node metastasis	12	11	>0.05

**Table 2:** Comparison of nutritional indexes between two groups.

	HGb (g/L)	ALB (g/L)	TP (g/L)	PA (mg/L)	TRF (mg/L)
Control group					
Before treatment	110.48±12.62	35.37±6.24	50.16±7.34	254.84±24.17	954.16±154.23
After treatment	120.23±18.50	40.71±4.14	57.31±6.68	270.63±18.55	2001.44±221.68
*t*	3.517	5.347	11.064	2.368	151.471
*P*	<0.05	<0.05	<0.05	<0.01	<0.01
Chinese herbal formula group					
Before treatment	110.24±5.47	36.62±4.50	49.67±7.45	262.47±25.39	975.51±183.17
After treatment	122.67±6.59	43.27±6.09	65.25±6.03	293.41±20.65	2517.54±208.61
*t*	2.647	6.382	10.930	3.417	184.173
*P*	<0.01	<0.05	<0.01	<0.01	<0.01

**Table 3:** Comparison of lymphocyte subsets between two groups before and after treatment.

	CD3+ (%)	CD4+ (%)	CD8+ (%)	CD4+/CD8+ (%)
Chinese herbal formula group				
Before treatment	53.34 ± 7.05	31.27 ± 5.40	36.21 ± 4.24	0.86 ± 0.22
After treatment	66.12 ± 5.68	40.22 ± 3.34	31.24 ± 5.37	1.29 ± 0.39
*t*	13.574	10.367	5.698	1.334
*P*	<0.01	<0.01	<0.01	<0.01
Control group				
Before treatment	53.15 ± 9.17	31.47 ± 6.25	36.93 ± 5.08	0.85 ± 0.11
After treatment	56.73 ± 6.46	35.04 ± 6.21	35.82 ± 3.63	0.98 ± 0.27
*t*	14.369	10.084	6.337	2.378
*P*	<0.05	<0.01	>0.05	<0.05

**Table 4:** Comparison of immunological indexes between two groups.

	IgG (g/l)	IgA (g/l)	IgM (g/l)
Chinese herbal formula group			
Before treatment	10.26 ± 1.05	2.27 ± 5.40	1.83 ± 4.24
After treatment	13.35 ± 5.68	2.95 ± 3.34	2.16 ± 5.37
*t*	0.444	0.286	0.559
*P*	<0.01	<0.01	<0.01
Control group			
Before treatment	10.37 ± 9.17	2.35 ± 6.25	1.79 ± 5.08
After treatment	11.50 ± 6.46	2.33 ± 6.21	2.09 ± 3.63
*t*	12.241	20.012	13.651
*P*	>0.05	>0.05	<0.05

**Table 5:** Comparison of TCM symptom score between two groups.

	*n*	Before treatment	After treatment
Chinese herbal formula group	33	32.52 ± 2.21	17.12 ± 2.58
Control group	33	33.02 ± 2.98	21.61 ± 1.36
*t*		1.472	3.635
*P*		>0.05	<0.05

**Table 6:** Comparison of adverse reactions between the two groups.

	*n*	Nausea and vomiting	Inappetence	Liver function impairment	Leukopenia	Thrombocytopenia	Total incidence (%)
Control group	33	4	3	2	3	4	48.5
Chinese herbal formula group	33	3	3	1	4	3	42.4

## Data Availability

The data used to support the findings of this study are available from the corresponding author upon request.
